# Will Improved Safety Attitudes Necessarily Curb Unsafe Behavior? Hybrid Method Based on NCA and SEM

**DOI:** 10.1155/2022/9271690

**Published:** 2022-09-16

**Authors:** Beifei Yuan, Shuitai Xu, Muqing Niu, Kai Guo

**Affiliations:** ^1^School of Economics and Management, Jiangxi University of Science and Technology, Ganzhou, Jiangxi 341000, China; ^2^First Affiliated Hospital, Henan University of Science and Technology, Luoyang, Henan 471003, China; ^3^School of Management, Henan University of Science and Technology, Luoyang, Henan 471003, China

## Abstract

As an inevitable product of the development of the construction industry, safety production has attracted more and more attention. In particular, it affects sustainable development. It is important to study the unsafe behavior of individuals. This study integrated the hybrid method of necessary condition analysis (NCA) and structural equation model (SEM). Based on the institutional environment perspective of social cognition theory, an empirical analysis was conducted through field observation and 186 questionnaire data to explore the influence of the institutional environment, safety attitude, and unsafe behavior. The results showed that improved safety attitudes of workers are a key requisite to curb unsafe behavior, and it was confirmed that safety attitude plays a complete mediating role between institutional environment and unsafe behavior. Through the analysis of the necessary conditions and mediating effects of safety attitude, the study deepened the theoretical understanding of the interaction between institutional environment, safety attitude, and unsafe behavior. Also, it provided relevant management suggestions for the construction industry in safety management.

## 1. Introduction

As a pillar industry in the world, the construction industry has more than 180 million employees and is expected to have a total output value of more than 1.05 billion in 2023, making a significant contribution to global economic development. With the continuous development of the construction industry, its safety production will still be a major problem troubling the healthy and sustainable development of the global economy [1]. Despite years of improvements in construction safety around the world, the construction industry is still statistically one of the riskiest in the world [2]. It accounts for about 30% of all industry deaths and has the second-highest rate of accidents among all industries [3]. Therefore, the government, society, and enterprises are deeply concerned about the problem of how to effectively prevent the construction industry production safety accidents. In recent years, academia and industry explore the causes of safety accidents; the analysis of safety accidents in the construction industry found that about 80% of the safety accidents were attributed to the unsafe behavior of construction workers [4]. Human safety attitude is an effective factor to predict unsafe behavior [5]; for example, a study of 500 workers found that people with a lack of safety attitudes were more likely to have accidents than others [6]. In the construction industry development wave, how to improve the safety attitude of construction workers, and then restrain the occurrence of unsafe behavior, has become a practical problem to be solved urgently in the construction industry. As an important phenomenon, safety attitude has also received widespread attention in academic circles [7].

At the macroenvironment level, the improvement of safety attitude includes profound changes in the engineering organization level of the entire project through changing the institutional environment [8]. At the microcognitive level, individuals' accident experiences can avoid unsafe behaviors by enhancing risk perception and improving safety attitude [9]. However, the research on safety attitude in relevant literature mainly focuses on the institutional environment or psychological cognition level, and the lack of the formation of safety attitude and its specific action mechanism on unsafe behavior is not conducive to the summary of management rules for the improvement of safety attitude. Safety behavior science is seen as the turning point of safety management research and brings new opportunities for safety science and safety psychology scholars [10]. Regarding the relationship between the institutional environment and unsafe behavior, safety behavior scientific literature generally starts from social cognition theory and finds that an institutional environment can promote individual safety attitude and safety behavior. For example, safety training can improve workers' risk identification ability [11]. In addition, safe construction can be effectively managed through a regulation system [12]. Many construction companies also began to improve the system environment, to achieve the improvement of workers' safety attitude and suppress the occurrence of unsafe behavior. These studies provide a useful reference in the article to explain the relationship between individual safety attitude and unsafe behavior from the perspective of the institutional environment.

Necessity and sufficiency are two different kinds of causality, which is the new focus of management research in recent years and the latest initiative of the chief editor of International Business Studies. Based on the institutional environment perspective of social cognition theory, this paper combines necessary condition analysis (NCA) and structural equation modeling (SEM). Analyzing the necessity and adequacy of institutional environment and individual safety attitude to unsafe behavior [13], this paper explores the complex process of how construction enterprises improve individual safety attitude and unsafe behavior by using the system. The problems to be solved include the following: (1) whether and to what extent safety attitudes are necessary to curb unsafe behavior? (2) Whether safety attitude mediates between institutional environment and unsafe behavior (i.e., safety attitude is a sufficient condition for unsafe behavior)? The possible research contributions of this paper include the following: first, it explains the internal mechanism of unsafe behavior from the perspective of the institutional environment and provides a different research perspective for safety management science in the study of unsafe behavior. Secondly, in the safety field, the hybrid method of NCA and SEM was used earlier to explore the relationship between the necessity and adequacy of safety attitude to unsafe behaviors, complementing the discussion on the adequacy conditions of variables by traditional regression research methods. Finally, this paper summarizes the antecedent and postpositional results of construction workers' safety attitudes from an empirical perspective and tries to further summarize the management rules of the formation and effect of safety attitudes, which is of great significance to help the construction party improve workers' safety attitudes and unsafe behaviors through the establishment of the institutional environment.

## 2. Theoretical Bases and Literature Review

### 2.1. Social Cognition Theory (SCT) and Institutional Environment Perspective

Social cognitive theory (SCT) has been widely used to explain the process of individual cognition to systematic behavior generation. According to this theory, individuals' behaviors are determined by the external environment and their own cognition [14]. The theory assumes that the environment, cognition, and behavior interact with each other. It emphasizes that individuals actively adjust their cognition to cope with changes in the external environment. Individual cognition determines behavior. Form a new feedback evaluation based on their individual situation environment. Therefore, individual cognition is influenced by the external environment, and then, this new cognition is transmitted to individual behavior.

In the field of organizational behavior, much literature finds that the institutional environment is fields that provides stable and normative cognitive structure and function for social behavior and can promote the stability of an individual or organizational behavior in the same field. The institutional environment is considered a “soft environment” that exerts a binding influence on an organization, including regulations, culture, and professional norms. In order to reduce the occurrence of total accidents in production, the construction companies need to form the system environment by integrating a regulation system, safety atmosphere, and safety training. However, the homogenization and ubiquity of best practices have led safety management scholars to question whether the institutional environment can directly affect individual unsafe behaviors [15]. Studies have found that the institutional environment often achieves intervention on unsafe behavior through other organizational factors. Existing studies believe that the isolated institutional environment does not have an impact and that it can only have an influence on individuals' attitudes when combined with individual cognition [16]. Therefore, although the institutional environment is a key resource, the inhibition of unsafe behavior is usually achieved by indirectly influencing individual cognitive factors.

Current studies generally adopt multiple dimensions to measure the institutional environment [8]. This paper explores the formation mechanism of unsafe behavior of construction workers from the perspective of the institutional environment of social cognition theory and draws on the research results of Mohammadi et al. [17], including regulatory system (RS), safety training (ST), and safety atmosphere (SA). Among them, the regulation system emphasizes that construction can effectively supervise construction workers to provide an excellent construction safety management system for construction workers. The safety training emphasizes that construction workers can carry out skill training to improve their professional quality and enhance their ability to deal with safety accidents. Safety atmosphere emphasizes that the construction group (such as workers) has good safety awareness towards safety construction.

### 2.2. Safety Attitude

The improvement of safety attitude is one of the main results of the improvement of the institutional environment. Improvement of safety attitude refers to the positive evaluation of individuals on the implementation of safety behaviors. In the construction site, improvement of safety attitude is defined as wearing safety hats when entering the construction site, placing construction tools in order, carrying out construction according to the safety process, and correcting the unsafe behaviors of workers around. Although organizations are constantly changing and developing to cope with the dynamic external environment, the improvement of safety attitude is based on the transformation of people's behavioral cognition, which has unique advantages in behavioral decision-making [18]. Concrete measures to improve safety attitude include integrating the system environment at the level of psychological cognition. Three environmental aspects are (1) corrective actions by managers, such as behavioral feedback and demonstration; (2) personal accident experience, such as accidents and risks experienced by workers in the past; and (3) safety skill training, such as regular communication of the key content of safe construction. The integration of these institutional environments and cognitive safety attitudes will form construction workers with safety attitudes [19]. Construction workers who combine the institutional environment with psychological cognition to improve their safety attitude would have great benefits in production safety [20]. A study of 636 construction workers at nine projects in Saudi Arabia found that construction workers with a good attitude toward safety were more likely than others to work safely [21]. The improvement of safety attitude has become one of the contents highly valued by the organization management. However, the existing research on how to implement a safety attitude promotion strategy is still scattered, mainly providing guidance for specific aspects of safety attitude [22]. Therefore, this paper is aimed at exploring how construction workers can improve their safety attitudes and further suppress unsafe behaviors through the institutional environment.

### 2.3. Unsafe Behavior

Due to the differences in research perspectives, the concept of unsafe behavior was not unified in the literature, and it was generally believed that unsafe behavior was the construction workers' violation of safety production system, safe operation methods, production technology regulations, and other behaviors that may cause safety accidents in the process of construction [23]. Choudhry [24] separated unsafe behaviors into two types: directly causing safety accidents and indirectly causing safety accidents. The direct type included failure to prevent hazard sources in time, such as entering the construction site with a risk of falling without a safety helmet. Indirectness mainly included not studying safety knowledge deeply. Martínez-Córcoles and Stephanou [25] further distinguished human subjective efficiency and divided unsafe behaviors into intentional violation type and unintentional cause type. Intentional violation type refers to the peculiar operation process of safe construction and the harm of unsafe construction but still uses unsafe behavior for construction. Intentional violation type refers to construction workers knowing the specific operational procedures of safe construction and the hazards of unsafe construction, but still adopt unsafe behaviors to carry out construction; unintentional causing type, refers to construction workers generally do not know enough about risk hazards and produce unsafe behaviors. Since this paper is aimed at highlighting the unsafe behavior of people, and the direct unsafe behavior can cause safety accidents at any time, it mainly focuses on the direct, intentional violation, and unintentional of these three aspects.

## 3. Research Hypotheses

### 3.1. Institutional Environment and Unsafe Behavior

Unsafe behavior is an obvious phenomenon but is affected by complex and changeable factors; the construction party needs to provide a good environment to realize the safe construction of construction workers, so as to avoid the occurrence of safety accidents. The institutional environment can help the construction party to integrate the internal and external environment, provide an environmental foundation for restraining unsafe behaviors, and effectively manage the specific process of safe construction, so as to ensure the safety of construction workers. For example, existing studies have found that builders can effectively manage the process of safe behavior, from job training to organizational institutionalization, using the institutional environment to improve worker safety behavior [26]. Fang et al. [27] took construction workers in Hong Kong as an example and found that regulation would directly affect the behavior of construction workers. Therefore, the institutional environment can effectively restrain unsafe behavior. Based on this, the following hypotheses are proposed:

*Hypothesis 1:* Institutional environment is negatively correlated with individual anxiety behavior (H1).

### 3.2. Institutional Environment and Safety Attitude

It is difficult for the constructors to restrain the unsafe behaviors of individuals by only relying on the intervention of the environmental level, while the transformation of the safety attitude at the psychological and cognitive level can realize the occurrence of safe behaviors of individuals. A recent study by Wang et al. [28] found that the institutional environment is, directly and indirectly, related to unsafe behaviors, especially that both are directly related to an individual's safety attitude, which in turn is related to unsafe behaviors. At present, the construction party needs to improve the safety attitude from the perspective of individual cognition to avoid unsafe behaviors. The improvement of safety attitude is the improvement of the construction party's regulation system, safety atmosphere, safety culture, and other environmental aspects, and it is a realization process from organizational management to individual management [8]. The basis of a safe attitude is the perception of risk, which then forms differentiated attitudes and behaviors. The improvement of safety attitude can promote the construction site to form a useful institutional environment and then promote construction workers to actively participate in safety construction activities. Current research also found that the institutional environment can further promote individual cognition, and a sound institutional environment can promote the improvement of individual safety cognition. For example, Warmerdam et al. [29] conducted research on 911 employees and found that in the absence of institutional supervision, employees mainly influenced their behaviors with their individual attitudes. In addition, the safety attitude needs multilevel intervention, including institutional supervision and safety atmosphere. Therefore, when the construction project has a high level of the institutional environment can effectively achieve a high level of safety attitude of construction workers and can realize the construction workers in accordance with the safety process. Based on this, the paper believes that the construction party has a higher level of institutional environment, more conducive to the improvement of individual safety attitude, and puts forward the following hypothesis:

*Hypothesis 2:* Institutional environment is positively correlated with the degree of individual safety attitude (H2).

### 3.3. Safe Attitudes and Unsafe Behaviors

Safety attitude reflects the construction workers' positive or negative evaluation of safety construction behavior and is the key factor to predict behavior intention. Henning et al. [30] argued that safety attitudes have differentiated effects among different individuals. To be specific, individuals selectively interpret the same situation differently according to their own preferences, and unsafe behaviors are not clearly defined in the formal rules of the organization, so there are differences among individuals. When the safety attitude is improved, it will also promote safety communication between individuals and project members, thus forming norms to further promote the safe construction of individuals. Man et al. [31] also confirmed this point of view by conducting a questionnaire survey of 536 construction workers and found that safety attitudes have a significant impact on safety behaviors. Timmermans et al. [32] found that continuous safety education and training can provide guidance for individual safety activities and help improve their safety attitude. Through the project team's safety communication, regulation system, and safety training, the construction site can form a good system environment, to achieve group safety construction. Based on the above key role of improving individual safety attitude in restraining unsafe behaviors, the following hypotheses are proposed from two aspects of necessity and adequacy:

*Hypothesis 3a:* The improvement of individual safety attitude is a necessary condition for inhibiting anxious behavior (H3a).

*Hypothesis 3b:* The improvement of individual safety attitude inhibits the generation of disquiet behaviors (H3b).

The exact research model and its hypothesis are shown in Figure 1.

## 4. Research Design

Sufficient and necessary causality are two different explanations of causality. In order to better analyze the complex causal mechanism of unsafe behaviors, SEM and NCA are, respectively, used in this study to verify the adequacy and necessity of research hypotheses. Considering that the partial least squares structural equation model (PLS-SEM) has advantages in exploratory research for theoretical development, analysis for prediction, and in the face of a complex structural model, can more effectively deal with nonnormal distribution data of questionnaire samples [33]. In addition, today's scholars often use the consistent PLS method for estimation. Its calculation method is the two-stage least squares method (2SLS), which can independently estimate each equation and is a technology with limited information. Therefore, PLS-SEM is used to test the adequacy of antecedent variables.

NCA is an emerging necessary condition analysis method. The necessary condition is that if a certain antecedent variable is missing in causality, the result cannot be realized. NCA is an effective supplement to the traditional regression analysis method (adequacy analysis) [13]. At the same time, the method can also quantitatively identify what degree of antecedent variables can achieve the necessary conditions of the results. Therefore, the NCA method is used to supplement the SEM method, and the effect size and bottleneck level of necessary conditions are analyzed.

### 4.1. Research Samples and Data Collection

#### 4.1.1. Unsafe Behavior Data Collection

In this study, the unsafe behavior data were collected by on-site observation. Through the field observation of 5 construction parties such as the First Construction Bureau of China Metallurgical Corporation and the Third Construction Bureau of China Construction Corporation in Ganzhou, Changsha, and Luoyang, the selected construction sites are all under construction and the number of project employees is not less than 70. A total of 10 construction projects are investigated to ensure the diversification of research data.

According to the accident investigation and the report of work Safety Administration Committee, the types of construction safety accidents are mainly composed of falling from a high altitude (53.69%), object strike (15.91%), earthwork, foundation pit collapse (8.93%), and lifting machinery injury (5.43%). Based on the above four main potential risks, combining reading-related academic literature [5], enterprise's safety management manual, and expert interview, the development of the construction workers' unsafe behavior observation scale, on this basis, to the construction site for field observation, understand the scene of each region of the work content and the type of work situation, and then, communicate and discuss with project management personnel of each site, revise the unsafe behavior scale of construction workers, and get the final list. The list mainly includes 14 unsafe behaviors in 4 categories, such as sitting in the area with falling risk, entering the site without wearing protective equipment such as a safety helmet, and removing formwork or support prematurely and a series of behaviors, as shown in Table 1. At present, most existing studies use self-reported questionnaires to measure unsafe behaviors of construction workers, which may lead to large measurement deviations [34]. Therefore, this study measures workers' unsafe and safety behaviors according to the observation scale “on-site observation,” and divides construction workers' safety behaviors into dichotomous variables “unsafe behaviors” and “safe behaviors, as shown below.

(1) $$\begin{array}{c} Y=\left\{\begin{array}{c} 1,\text{workers were observed to exhibi}{\text{t}}^{"}\text{unsafe behavior}{,}^{"}\\ 0,\text{other }\left(\text{safety behavior}\right), \end{array}\right. \end{array}$$

where *Y* = 1 indicates that the worker's behavior is unsafe and *Y* = 0 indicates that the worker's behavior is safe.

The specific experiment is as follows: firstly, 15 observers with rich construction experience are selected, and case samples of workers with unsafe behaviors are selected according to the unsafe behavior observation scale on site. Before starting the survey, the observers informed each construction worker that the purpose of the study was academic research, that there was no business relationship with the construction party, and that the results of the survey would help the construction workers win the support of the construction workers in a safer working environment by eliminating their doubts. Secondly, considering that the presence of observers may lead to behavioral deviation of workers, observers are required to observe and record as far as possible in the first site. It is found that people's potential behavioral deviation for the presence of observers is reduced, the behavioral deviation is normalized, and the handling method is recognized by the person in charge of the site. Finally, the recorded observations were matched with the questionnaire results of the same construction worker.

#### 4.1.2. Descriptive Statistical Analysis

A total of 200 questionnaires were sent out in the study, with an average of 20 for each site. A total of 186 valid questionnaires were collected, with an effective recovery rate of 93%, excluding those with incomplete interviews and chaotic logical expression. The sampling process can be considered as simple random sampling because construction workers are selected by random observation in the project. The descriptive statistical consequences of the respondents are shown in Table 2. Local construction workers are predominantly male, in line with the actual situation on construction sites. The age distribution of the samples was less than 25 years old, 12.8%; 25-35 years old, 23.8%; 35-45 years old, 32.9%; and over 45 years old, 30.5%. Construction workers over 35 years old accounted for 63.4%, in line with the “aging” population characteristics of today's construction sites. Most of the workers' education level is lower than that of senior high school (68.9%), which also shows the reality that the construction workers' education level is not high. Among them, most of the workers have more than 10 years of work experience, accounting for 60.4%, indicating that the respondents have relatively rich work experience. In addition, the distribution of various types of work is relatively uniform.

This paper uses the method of comparing the questionnaire of construction workers before and after the survey to check whether there is no response error in the sample. Statistical results show that there is no significant difference between the two groups of samples in the variables of job type, working years, education level, and so on (*P* > 0.1), so there is no problem of response error in the study.

### 4.2. Variable Measurement

The questionnaire mainly measures the institutional environment (including institutional control, safety training, and safety atmosphere) and safety attitude. In order to ensure the reliability and validity of the questionnaire, the variables were measured by referring to the existing maturity scale and combining it with the safety practice of Chinese construction enterprises. For English questions, the study followed translation and back translation procedures to ensure the accuracy of questionnaire translation. The questionnaire used a five-point Likert scale. In addition, prior to the formal investigation, construction workers on the construction site should be presurveyed, and the questionnaire should be adjusted accordingly according to the feedback obtained from the presurvey, so as to ensure the clear expression of the questionnaire. Specific index items are shown in Table 3.

The institutional environment reflects the construction party's safety resource conditions and the degree of support for safety management. Based on existing studies [35], the institutional environment of the paper includes three dimensions: institutional control, safety training, and safety atmosphere. Among them, the regulation system emphasizes that the construction party can carry out effective supervision and reward and punishment intervention on workers, mainly including safety assessment and on-site supervision and other three indicators to measure. Safety training focuses on the construction party's ability to build worker safety capacity with available resources in advance, which is measured using three indicators. A safety atmosphere emphasizes the attitude of construction team members towards safe construction, and four indicators are used to measure it.

Safety attitude refers to the scale of existing studies [36], which reflects the individual's value judgment and emotional color of safety, namely, an individual's view of safe construction. Based on the practice of construction enterprises in China, the Delphi method was used to score the items iteratively, and finally, three indexes of safety attitude were determined.

Furthermore, we took the individual characteristics of unsafe behaviors (work experience, educational background, and job category) as control variables. Among them, all control variables are represented by fixed class variables in Table 2.

## 5. Data Analysis

### 5.1. Measurement Model Analysis

In this study, SPSS 24.0 was utilized and used to test the reliability of the sample data. Firstly, the reliability of the overall questionnaire was analyzed, and the Cronbach's *α* value of the overall questionnaire was 0.861, indicating that the overall reliability of the questionnaire was good. The reliability analysis of different variables showed that Cronbach's *α* value of each variable was between 0.804 and 0.875, which met the threshold of Cronbach's *α* value greater than 0.7, showing that the survey measurement item has high reliability and can reflect each variable accurately [37, 38]. The validity was further tested. Firstly, the KMO test and Bartlett test were carried out on the questionnaire, and the KMO value was 0.823, higher than 0.8, and the significance (*P* ≤ 0.001) was less than 0.05, so it was suitable for factor analysis. In the validity test, convergence validity and discriminant validity were used to access the comprehensiveness and exclusivity of variables, respectively. Convergence validity was tested by the mean-variance extraction (AVE), combined reliability (CR), and factor loading of latent variables. The measurement variables are required to correspond to factor loading values greater than 0.6 and CR values greater than 0.7. The factor load values in the study all ranged from 0.543 to 0.942 (Table 4), and CR values of all variables were greater than 0.7 (Table 3), indicating that each dimension had high internal consistency. Among them, the acceptable range of AVE value is 0.36~0.50, and greater than 0.5 are ideal. AVE values of all variables in the study are greater than 0.5 (Table 4), indicating that the study dimension can explain the variance of variables well and has good convergence validity.

The discriminant validity test should meet the requirement that the AVE square root of all variables is larger than the correlation coefficient between the variable and other variables. The italic part in Table 4 is the AVE square root of each variable. It is found that the correlation coefficients of the 5 research variables all meet the requirements.

### 5.2. Structural Model Analysis

The structural model analysis results of the individual unsafe behavior research model are shown in Figure 2. Structural model analysis is mainly evaluated from four aspects: SRMR, *R*^2^, path coefficient, and significance. The SRMR value of the model studied in this paper is 0.064, lower than the standard of 0.08, so it meets the requirements of model fit of PLS-SEM. *R*^2^ of unsafe behavior and safety attitude was 0.294 and 0.378, respectively, indicating that the variance explanation rate of unsafe behavior and safety attitude was 29.4% and 37.8%. It meets the *R*^2^ threshold requirements proposed by Hair et al. [33].

### 5.3. Common Method Deviation Test

In order to improve the effectiveness of the case, the following measures are taken to avoid common method errors: (1) inform workers in advance that the research is academic only. (2) Interview results will be anonymized. (3) Interview questions should be concise and easy to understand. (4) Set some reverse items, and measure at a different time and other facilities to control the common method deviation from the program. After obtaining the data, we used the Harman single-factor method to test the common method bias. In the factor analysis without rotation, a total of 4 principal components with eigenvalues greater than 1 were extracted. The maximum principal component explained 32.11% of the total variance, which was far lower than 40% of the threshold standard [39]. Therefore, the common method bias in this study is within an acceptable range.

### 5.4. Hypothesis Testing of Necessity and Adequacy

As for the necessity analysis of antecedent variables, this study uses the NCA package of R software to test the necessary of institutional control, safety training, safety atmosphere, safety attitude, and unsafe behavior, respectively. Firstly, the upper bound function is determined for effect value analysis of antecedent variables, and ceiling regression (CR) and ceiling envelope (CE) methods are usually used to select the upper bound function, wherein the CR method is suitable for processing continuous variables and discrete variables. CE method deals with 2 score variables or discrete variables less than 5.

In Table 5, NCA analysis results are reported, including the use of CR and CE to calculate the effect size and *P* value, to improve the robustness of the results. The results show that the improvement of a safety attitude is a necessary condition to suppress unsafe behaviors, and the effect values (*d*) are above 0.1, which belongs to the medium level. Monte Carlo simulation of permutation tests also reaches a significant level. However, the results of institutional regulation (*P* = 1.0), safety training (*P* = 1.0), and safety atmosphere (*P* = 1.0) were not significant, indicating that they are not necessary conditions for restraining unsafe behaviors.

The bottleneck analysis results are reported in Table 6. The bottleneck level value is a level that reaches the maximum observation range of the effect and the level value that needs to be satisfied within the maximum observation range of the variable. The results show that an 11.2% safety attitude is needed to restrain 60% of unsafe behaviors, and there is no bottleneck level in institutional control, safety training, and safety atmosphere. So H3a is supported.

Smart PLS 3.0 software was used in this study to analyze the adequacy of antecedent variables. In order to ensure the consistency of computation, the path coefficients and statistical significance were analyzed by combining the consistent PLS algorithm with the bootstrapping method of 5000 times resampling. The structural model analysis results of the unsafe behavior research model are shown in Figure 2.

Three control variables (educational background, working time, and job type) have no significant influence on unsafe behavior. The results show that all three theoretical hypotheses are valid at the significance level of 5%, as shown in Figure 2. Specifically, the institutional environment has a significant negative impact on unsafe behavior (*β* = −0.339, *P* ≤ 0.01), H1 verified; institutional environment significantly positively affected safety attitude (*β* = 0.278, *P* ≤ 0.01), verified for H2; safety attitude significantly negatively affected unsafe behavior (*β* = −0.202, *P* ≤ 0.05), assuming that H3b is true.

### 5.5. Intermediate Inspection

Analysis of the mediating effect of safety attitude: referring to the suggestions, Liu et al. [40] verify the mediation effect of the three conditions: (1) the coefficient of the dependent variable (DV) is significant in the regression of the independent variable (IV). (2) The coefficient of the dependent variable is significant in the regression of the intermediate variable (M). (3) When the dependent variable is regressive at the same time between the mediation variable and the independent variable, the coefficient is significant. If the independent variable coefficient is larger in the case of (1) than (3), there is a complete mediation effect. The mediating effect analysis in Table 7 (from columns 4 to 6) shows that a safety attitude completely mediates the relationship between the institutional environment and unsafe behavior. Meanwhile, the bootstrap method (*N* = 5000) is used to test the mediation effect. The process program issued by SPSS software is used to test the confidence interval (BootCL upper and lower limits) generated by SPSS (Table 7). If there is no 0 between BootCL upper and lower limits, it indicates that the mediation effect is significant. According to Table 7, the 95% error correction interval for 5000 samples is calculated, which does not contain 0. These results further confirm that safety attitude plays a mediating role in the relationship between the institutional environment and unsafe behavior.

## 6. Research Conclusions and Implications

### 6.1. Research Conclusions

Based on the institutional environment perspective of social cognition theory, this study investigated 186 construction workers and found that the institutional environment had a positive effect on unsafe behavior and safety attitude, while safety attitude had a negative effect on unsafe behavior. Among them, the improvement of safety attitude is the necessary condition of unsafe behavior and plays a complete mediating effect between institutional environment and unsafe behavior. This study deepens the theoretical cognition of the relationship between institutional environment, safety attitude, and unsafe behavior and provides a useful reference for the safety management of the construction industry. The main conclusions are as follows:

First, the institutional environment of the project is measured from three dimensions of institutional control, safety training, and safety atmosphere, and the positive effect of the institutional environment on safety attitude and unsafe behavior is verified by a second-order model. Existing studies quantify unsafe behavior mainly through questionnaire measurements of workers, and it is difficult to measure the real data on unsafe behavior. In this paper, the data on unsafe behavior is measured by on-site observation. This paper uses the data of construction workers to verify the effectiveness of the institutional environment from three dimensions of the institutional environment, safety training, and safety atmosphere and the positive effect of the institutional environment on safety attitude and unsafe behavior.

Secondly, according to the empirical data of construction workers, it is verified that safety attitude plays a complete intermediary effect between institutional environment and unsafe behavior, and the specific mechanism of institutional environment on unsafe behavior is improved. Existing studies mainly discuss the role of the environment on unsafe behaviors, but the lack of discussion on specific processes (such as ignoring the role of safety attitudes). Based on the perspective of the institutional environment, this study adopts a quantitative research method to explain the mechanism of the institutional environment promoting safety attitude and inhibiting unsafe behavior.

Finally, using NCA's necessary conditions analysis, it was found that safety attitude enhancement is a necessary condition and an important bottleneck to curb unsafe behavior. At present, there are few types of research on necessary conditions in safety management literature, and the research on safety attitude and unsafe behavior is mainly based on the sufficient condition test of the traditional regression method. Therefore, the combination of NCA and SEM in this study is conducive to promoting the development of research on the necessary and sufficient relationship between safety attitude and unsafe behavior.

### 6.2. Theoretical Enlightenment

This paper also has some theoretical contributions to safety management literature, mainly including the following two aspects:

First, the institutional environment for on-site safety management and the occurrence of unsafe behaviors has aroused the widespread attention of scholars today [41]. From the perspective of the institutional environment, this paper can effectively integrate the relevant research results of institutional environment and safety attitude and explain the internal mechanism of individual safety attitude restraining unsafe behaviors from the perspective of psychological cognition, providing a new research perspective for safety management scholars to study behavior safety management at the micro institutional level.

Second, in the field of safety, the necessity and adequacy of improving safety attitude are comprehensively discussed by using the hybrid research method combining NCA and SEM earlier. In particular, through the identification of the necessary conditions for "safety attitude enhancement", the article is of great theoretical significance for the construction side to optimize the relevant safety attitude enhancement strategies, so as to ensure that the safety attitude enhancement of construction workers is at the "appropriate level and above" and thus inhibit the occurrence of unsafe behaviors. It has important theoretical significance.

### 6.3. Management Implications

This paper has significant management enlightenment for the construction party to improve the institutional environment and improve the safety attitude of construction workers. First of all, in terms of organizational culture construction, the improvement of personal safety attitude requires the construction party to create an excellent institutional environment, which mainly includes institutional control, safety training, and safety atmosphere. The construction party needs long-term investment and construction in the three aspects to realize the improvement of construction workers' safety attitude. For example, on the construction site, actively promote safety training activities, full participation in safety activities, and the implementation of safety reward and punishment strategies for employees, and actively promote the improvement of construction workers' safety attitude. Secondly, in terms of safety management, the improvement of construction workers' safety attitude is the only way the development of safety management. Therefore, the construction party should pay attention to the important role of personal safety attitude in safety management, and actively use the institutional environment and other organizational resources to jointly promote the improvement of personal safety attitude (such as VR accident experience and eye-tracking study), so as to realize safety management and intelligent implementation and also promote the transformation and upgrading of the traditional construction industry [42]. Finally, the construction party should actively build the safety culture of the project, and create a positive safety culture which is the embodiment of effective safety communication among team members, and then affect the safety atmosphere of the team, and correct the unsafe attitude of construction workers, so that safe construction in the project becomes a normal state.

### 6.4. Limitations and Future Directions

The article also has some limitations, which need to be further improved in the future: (1) as for the causes of the improvement of safety attitude, this paper mainly starts from the perspective of the institutional environment. In fact, other influencing factors will also affect the improvement of safety attitude, such as the influence of employees' families [43]. Future studies can incorporate these factors into the model. (2) Avoiding a single data source, this paper analyzes the relationship between the institutional environment, improvement of safety attitude, and unsafe behavior with cross-sectional data from field observation and questionnaire data. In the future, the causal relationship among variables will be further studied from the perspective of dynamic evolution. (3) NCA and SEM are utilized used to analyze the necessity and adequacy of a single variable. Further studies on the adequacy of combinations of different antecedents can be carried out from a configuration perspective in the future.

## Figures and Tables

**Figure 1:** Research hypothesis model.

**Figure 2:** Structural model results.

**Table 1:** Safety observation scale for construction worker behavior.

No.	Type of accident risk	Specific unsafe behaviors
1	High falling	Sitting in areas at risk of falling (such as railings and scaffolding.)
		Using incorrect climbing tools (such as material lifting device)
		In the process of erecting scaffolding and steel support, the platform is unsafe and no safety belt is used
		Unauthorized removal of safety protection devices
2	Object strike	Personal protective equipment such as safety hats not worn on the site
		Transmission of tools and materials at high places
		No safe passage on construction site
3	Earth, foundation pit collapse	Safety measures such as premature removal of formwork or support
		Entering the pit from the edge of the pit with large slopes or obstacles
		Do not set up scaffolding as required
4	Lifting machinery damage	Wearing gloves to command or operate slings, or multiple people to command, without standard gestures
		The lifting operation through the personnel area or the operation area does not ring the flute
		Maintenance, cleaning, maintenance, and so on during mechanical operation

**Table 2:** Demographic characteristics of construction workers (*N* = 186).

Characteristics	Number	Percentage (%)
Gender		
Male	141	75.8
Female	45	24.2
Age		
<25 years	26	14
25~35 years	44	23.7
35~45 years	60	32.3
>45 years	56	30.1
Work experience		
<5 years	23	12.4
5~10 years	52	28
10~15 years	55	29.6
>15 years	56	29.6
Educational background		
Primary school or below	51	27.4
Secondary school	74	40
Senior high school	39	21
Bachelor's degree and above	22	11.8
	
Job category		
Steel fixer	50	26.9
Solid plasterer	31	16.7
Scaffolder	38	20.4
Special type operator	50	26.9
Others	17	9.1

**Table 3:** Construct measurement and convergent validity analysis.

Construct	Indicator	Variable description	Standardized loading	AVE
Regulation system (RS)	RS_1_	The company will regularly organize security assessments	0.908	0.713
	RS_2_	If I do not have protective equipment, my supervisor will scold me	0.873	
	RS_3_	Safety guards supervise staff behavior at the construction site	0.743	
Safety training (ST)	ST_1_	My company trains employees on workplace safety issues	0.836	0.792
	ST_2_	Give me safety training enough to assess workplace hazards	0.840	
	ST_3_	Management encourages us to attend security training courses	0.744	
Safety atmosphere (SA)	SA_1_	Management takes corrective action against unsafe measure	0.654	0.594
	SA_2_	Team members provide guidance for security work	0.876	
	SA_3_	Team members remind the use of safety equipment	0.864	
	SA_4_	Team members discuss security risks	0.657	
Safety attitude (SA)	SA_1_	Accidents at work are inevitable	0.845	0.766
	SA_2_	I can also do the work of security personnel, which is relatively simple	0.924	
	SA_3_	If the safe operation rules are convenient and feasible, it can promote my safe work	0.855	

**Table 4:** Mean, standard deviation, correlation coefficient, and discriminant validity.

Variable	IE	SA	USB	EB	WE	JC
Institutional environment	*0.748*					
Safety attitude	0.221^∗∗^	*0.875*				
Unsafe behavior	-0.342^∗∗^	-0.302^∗∗^	*1*			
Education background	-0.154	-0.040	-0.029	1		
Work experience	0.010	-0.066	-0.208^∗∗^	0.042	1	
Job category	0.018	-0.102	0.240^∗∗^	-0.237^∗∗^	0.048	1
Mean	3.849	3.369	0.500	2.130	2.740	2.800
Standard deviation	0.679	1.255	0.502	0.931	1.362	1.003

Note: ^∗^*P* ≤ 0.05; ^∗∗^*P* ≤ 0.01; the italic part of the diagonal is the AVE square root.

**Table 5:** NCA method necessary condition analysis results.

Variables	Method	Accuracy	Ceiling zone	Scope	Effect of value (*d*)	*P* value
Regulation system	CR	100%	0.000	4.00	0.000	1.000
	CE	100%	0.000	4.00	0.000	1.000
Safety training	CR	100%	0.000	4.00	0.000	1.000
	CE	100%	0.000	4.00	0.000	1.000
Safety atmosphere	CR	100%	0.000	4.00	0.000	1.000
	CE	100%	0.000	4.00	0.000	1.000
Safety attitude	CR	100%	0.023	4.00	0.000	0.001
	CE	100%	0.037	4.00	0.140	0.001

Note: d: 0.0 ≤ d < 0.1 is the low level and 0.1 ≤ d < 0.3 is the medium level; P: substitution test for NCA analysis (permutation test, *N* = 10000).

**Table 6:** NCA method bottleneck level (%) analysis results.

Curb levels of unsafe behavior	Regulation system	Safety training	Safety atmosphere	Safety attitude
0	NN	NN	NN	NN
10	NN	NN	NN	NN
20	NN	NN	NN	NN
30	NN	NN	NN	NN
40	NN	NN	NN	NN
50	NN	NN	NN	5.2
60	NN	NN	NN	11.2
70	NN	NN	NN	17.1
80	NN	NN	NN	23.1
90	NN	NN	NN	29.0
100	NN	NN	NN	35.0

Note: NN: unnecessary.

**Table 7:** Analysis of the mediating effect of safety attitude.

X + M → Y							Bootstrap analysis			
X	M	Y	X → Y	X → M	X	M	Mediation effect	BootCL min	BootCL max	Intermediation
IE	SA	USB	-0.254^∗∗∗^	0.407^∗∗^	0.415^∗∗∗^	-0.420^∗∗∗^	-0.174^∗∗∗^	-0.405	-0.034	Full mediation

Note: ^∗∗∗^*P* ≤ 0.001 and ^∗∗^*P* ≤ 0.01.

## Data Availability

The data used to support the findings of this study are available from the corresponding author upon request.
